# Effect of Chronic Heart Failure Complicated with Type 2 Diabetes Mellitus on Cognitive Function in the Elderly

This article has been retracted.

**DOI:** 10.1155/2022/4841205

**Published:** 2022-06-28

**Authors:** Yang Liu, Rui Meng, Jianzeng Dong

**Affiliations:** ^1^Department of Cardiology, Anzhen Hospital, Capital Medical University, Beijing 100029, China; ^2^Department of Geriatrics, Aerospace Center Hospital, Beijing 100029, China

## Abstract

**Objective:**

To explore the effect of chronic heart failure complicated with type 2 diabetes mellitus on cognitive function in the elderly.

**Methods:**

600 patients with chronic heart failure were selected from January 2018 to January 2021. All patients were divided into observation group (A) and control group (B). A was chronic heart failure complicated with type 2 diabetes mellitus group. B was chronic heart failure group. The clinical effects of the two groups were observed.

**Results:**

Compared with the clinical indexes during and after operation, there were differences in operation time, postoperative recovery time, and treatment cost between A and B, but the difference is not significant (all *P* > 0.05). LVEF cardiac function index score, LVEF score of A compared with B, the difference was statistically significant (*P* < 0.05). The MMSE score and MoCA score of the two groups were compared. Before operation, the MMSE score and MoCA score of A were lower than those of B, and the difference was statistically significant (*P* < 0.05). After operation, the MMSE score and MoCA score in B were significantly higher than those in B, but the increasing trend of MMSE score and MoCA score in B was significantly higher than that in A (*P* < 0.05). Comparison of HAMA score and HAMD score: before operation, the HAMA score and HAMD score were higher in A, but the difference is not significant (*P* > 0.05). After operation, the scores of HAMA and HAMD in A and B decreased significantly, but the difference is not significant (*P* > 0.05). Multivariate analysis showed that the fasting blood glucose and glycosylated hemoglobin were the risk factors of cognitive impairment.

**Conclusion:**

Type 2 diabetes mellitus in elderly patients with chronic heart failure will further aggravate cognitive impairment, and type 2 diabetes is an important independent risk factor affecting cognitive function, which accelerates cognitive impairment and significantly reduces the executive ability of elderly patients with chronic heart failure, resulting in a significant decline in patients' ability to understand and apply information.

## 1. Introduction

Chronic heart failure (CHF) is a serious stage in which hypertension, coronary heart disease, cardiomyopathy, and other cardiovascular diseases develop to the end stage [1, 2], which is mainly caused by cardiac pumping dysfunction, and has the characteristics of complex, chronic, recurrent attacks, and so on [3–5]. CHF often occurs among the middle-aged and elderly [6]. On account of the development trend of aging in recent years, the number of patients with this disease has increased year after year, and the number of CHF patients worldwide has reached 11 million [7]. Previous studies had also shown that there is a close relationship between CHF and cognitive function, and more and more studies have confirmed that CHF patients are more likely to develop cognitive impairment (CI) [8]. CI mainly refers to memory disorders, aphasia, visual-spatial disorders, executive dysfunction, dyscalculia, apraxia, agnosia, and dementia. Concomitant symptoms also include sensory disorders, thinking disorder, affective disorder, and will and behavior disorder. Therefore, clinicians pay more and more attention to the cognitive function of patients with CHF [9, 10].

Some clinical data also show that there is serious cognitive impairment in senile CHF itself, and diabetes is the main factor in the development of CHF, and type 2 diabetes mellitus (T2DM) is especially common in CHF patients with CI [11–13]. The mortality caused by the combination of the two is higher than that in nondiabetic patients, which further aggravates the cognitive impairment, increases the hospitalization rate and mortality, and the quality of life of patients is seriously affected [14, 15]. However, some studies have found that type 2 diabetes is the main factor leading to dementia and cognitive impairment in patients with CHF, and type 2 diabetes is likely to be an independent risk factor for CI [16]. Therefore, for the elderly CHF patients with T2DM, we should be concerned about the effect of blood glucose levels on the cognitive function of the elderly and closely monitor the blood glucose of the patients [17].

As the elderly suffer from chronic diseases, they also suffer from CHF and diabetes. Most studies show that the rate of cognitive impairment is as high as 75%–80% [18]. 25%–75% of CHF patients have serious cognitive impairment, which seriously threatens the quality of life of the elderly, resulting in lower compliance and lower self-care ability. Increased readmission and mortality [19]. This study is a retrospective study of elderly patients with cognitive function and explores the clinical observation of the effect of CHF combined with type 2 diabetes on the cognitive function of the elderly so as to prevent and delay the development of CI in the early stage, further improve the prognostic of patients with CHF, and improve the quality of life of the elderly.

## 2. Methods

### 2.1. Study Design and Participants

A total of 600 patients with CHF treated in Anzhen Hospital of Capital Medical University from January 2018 to January 2021 were selected. All patients were divided into the observation group (A, *n* = 306) and control group (B, *n* = 337), 152 males and 154 females, aged 60–94 years, and 165 males and 172 females, aged 60–94 years. There was no difference in the condition, course of the disease, and other general data of the selected patients (*P* > 0.05), which was comparable. All the subjects obtained informed consent. The study was approved by the Anzhen Hospital Ethics Committee (No. AZ2912). All participants had a complete medical history examination and clinical examination.

### 2.2. Observation Index

(1) Comparison of clinical indexes: the operation time, postoperative recovery time, treatment cost, and left ventricular ejection fraction (LVEF score) of the three groups were recorded. LVEF is one of the most commonly used indicators of cardiac function. The recovery of cardiac function of the two groups was judged by measuring the percentage of LVEF. Clinical data show that LVEF can also reflect the cognitive function of patients.
(2) MMSE (Terrier cognitive assessment scale) score and MOCA (Montreal Cognitive Assessment Scale) score were used to score the cognitive work of the two groups. The cognitive work scores of the patients before and after the operation were observed and compared:
  ① The MMSE test includes language, immediate memory, reading comprehension, language comprehension, short-term memory, language retelling, naming objects, and other scores. The full score is 30, the higher the score, the better, and more than 24 indicates that the cognitive function is normal.
  ② The MoCA test includes visual space and executive function, naming, memory, attention, language, abstract understanding, delayed recall, orientation, and other items. The full score is 30, the higher the score, the better, and more than 26 indicates that the cognitive function is normal.
(3) HAMA (Hamilton Anxiety Scale) score and HAMD (Hamilton Depression Scale) score were used to score the degree of anxiety and depression of the two groups. The preoperative and postoperative anxiety and depression scores were observed and compared: HAMD and HAMA scales include 24 items and 14 items respectively. The higher the total score, the more serious the anxiety and depression.
(4) The related OR and *P* values were measured, and the effect of type 2 diabetes on cognitive function was studied by Logistic regression analysis.

#### 2.2.1. Inclusion and Exclusion Criteria

Inclusion criteria are as follows: (1) suffered from CHF and was diagnosed with CHF. (2) The age is not less than 60 years old. (3) There is no mental illness and no long-term use of psychotropic drugs. (4) Patients actively participate, and all patients sign informed consent. Exclusion criteria are as follows: (1) complicated with other severe acute cardiovascular and cerebrovascular diseases. (2) Unconscious or severe mental illness. (3) Neurological diseases that may affect cognitive function, such as dementia. (4) Addiction to psychoactive substances.

### 2.3. Statistical Analysis

This is a retrospective study. The data were statistically processed by the SPSS26.0 software, the measurement data were expressed as median, the differences between groups were compared by the *t*-test, and the counting data were expressed by frequency and *X*^2^ test. Logistic regression was used to analyze the risk factors of cognitive impairment, with *P* < 0.05 as the difference, which was statistically significant.

## 3. Result

A total of 643 elderly patients with CHF complicated with type 2 diabetes mellitus in our hospital from June 2018 to June 2021 were selected, including 306 patients in the A group and 337 patients in the B group. There were 152 males and 154 females in the A group, aged from 60 to 94 years old, with an average age of 78.2 ± 8.5 years and BMI of 24.39 ± 1.73. The patients in the B group included 165males and 172females, aged from 63 to 88 years old, with an average age of 77.9 ± 7.8 years and BMI of 24.63 ± 1.51. There was no difference in the condition, course of the disease, and other general data of the selected patients, *P* > 0.05, Table 1.

### 3.1. Comparison of Clinical Indexes during and after Operation

LVEF is one of the most commonly used indexes to judge cardiac function. The LVEF score of the A group was lower than that of the B group (*P* < 0.05), Table 2.

### 3.2. Comparison of MMSE Score and MOCA Score

Before the operation, there was no significant difference in MMSE score and MoCA score between the A group and B group (*P* < 0.05). After the operation, compared with the B group, the MMSE score and MOCA score in the A group were significantly higher, but the rising trend of MMSE score and MOCA score in the B group was significantly higher than that in the A group (*P* < 0.05), Table 3.

### 3.3. Comparison of HAMA Score and HAMD Score

Before the operation, there was no significant difference in the HAMA score and HAMD score (*P* > 0.05). After the operation, the scores of HAMA and HAMD in the A group and B group decreased significantly, But the difference is not significant, Table 4.

### 3.4. Multivariate Analysis of Risk Factors Leading to Cognitive Dysfunction

The OR values of fasting blood glucose and glycosylated hemoglobin were more than 1 (*P* < 0.05), so it was considered to be the risk factor for cognitive dysfunction, Table 5.

## 4. Discussion

CHF is a syndrome of cardiac insufficiency caused by various heart diseases [20]. The main clinical manifestations are dyspnea, fatigue, pulmonary congestion, and systemic blood stasis, which is an irreversible process of chronic disability and needs long-term treatment [21]. Diabetes is the most common chronic metabolic disease, which can lead to serious complications of heart, brain, kidney, blood vessels, nerves, and other tissues and organs [22]. Elderly patients with CHF with diabetes are a special group, which is a serious threat to human health [23]. Previous studies have shown that diabetes can lead to sympathetic dysfunction through metabolic and hemodynamic factors, which further lead to the decrease of the bioavailability of nitric oxide and the increase of protein kinase c13 expression [24, 25], and superimposed with diabetic hyperglycemia and insulin resistance, resulting in serious damage to endothelial function, reduction of myocardial blood supply, and the gradual formation of chronic heart failure [26].

CHE is a common disease in elderly patients in the department of cardiology, which has the characteristics of complex, chronic and recurrent attacks, and often occurs in middle-aged and elderly people [27–29]. With the aggravation of the aging problem of the population, the number of patients with this disease is increasing year after year, and the incidence of CHF is also gradually increasing. In recent years, studies at home and abroad have shown that there is a close relationship between CHF and cognitive function, and there is a serious cognitive impairment in CHF itself [30]. Some studies have shown that diabetes is the main cause of clinical symptoms of heart failure [31, 32]. The incidence of CHF in diabetic patients is more than 10%, which increases the mortality and disability rate of patients. The mortality caused by the combination of them will be about 8 times higher than that of nondiabetic patients [33]. Diabetes, as the main high-risk factor for aggravating CHE, increases the risk of cognitive impairment and dementia to some extent [34]. The quality of life of the patients was seriously affected to further aggravate the degree of cognitive impairment, increase the hospitalization rate and mortality, and the prognosis was very poor [35]. With the increase in blood glucose, the process of protein glycation is enhanced and the end products of irreversible glycation are produced too much. The formation of advanced glycation end products changes the structure, physicochemical properties, and functional state of the protein. Other studies have shown that long-term hyperglycemia can cause chronic diabetic encephalopathy. It may also cause peripheral microvascular complications. Because diabetic microvascular complications are the characteristic pathological damage of diabetes, the cognitive function of patients with microvascular complications is significantly lower than that of patients without complications. This suggests that the decline of cognitive function in patients with diabetes is related to diabetes itself. Chronic heart failure and diabetes are two major epidemics in modern times, both of which occupy a considerable proportion of medical resources around the world [36, 37]. It has become a public health problem that has been paid close attention to at home and abroad. The diagnosis and treatment of elderly patients with chronic heart failure complicated with type 2 diabetes mellitus is also the focus of clinical research [38].

The results of this study showed that there were differences in operation time, postoperative recovery time, and treatment cost between the A group and B group, but the difference is not significant(all *P* > 0.05). Clinical data showed that LVEF can reflect the cognitive function of patients. Through the LVEF cardiac function score of the two groups of patients, it was found that the difference of LVEF scores between the A group and B group was statistically significant (*P* < 0.05), indicating that patients with type 2 diabetes had poor recovery of cognitive function after the operation. Type 2 diabetes is an independent risk factor affecting the cognitive function in the elderly. Compared with the B group, the MMSE score and MOCA score in the A group were significantly higher, but the rising trend of MMSE score and MOCA score in the B group was significantly higher than that in the A group (*P* < 0.05). The HAMA score and HAMD score in the A group and B group were significantly lower than those in the B group, and the difference is not significant(*P* > 0.05). Logistic multivariate analysis showed that fasting blood glucose and glycosylated hemoglobin were the risk factors of cognitive impairment.

Based on the above conclusions, chronic heart failure complicated with type 2 diabetes is very common in clinic. The clinical symptoms of patients with codisease are more severe, and the prognosis is worse than those with single disease. Type 2 diabetes mellitus in elderly patients with chronic heart failure will further aggravate cognitive impairment, and type 2 diabetes is an important independent risk factor affecting cognitive function, which accelerates cognitive impairment and significantly reduces the executive ability of elderly patients with chronic heart failure, resulting in a significant decline in patients' ability to understand and apply information. To sum up, great attention should be paid to whether the elderly with chronic heart failure have type 2 diabetes or not.

## Figures and Tables

**Table 1:** Baseline characteristics of participants.

	A group (*N* = 306)	B group (*N* = 337)
Gender (male/female)	152/154	165/172
Age (*x* ± *S*, years)	78.2 ± 8.5	77.9 ± 7.8
Weight (kg)	65.7	67.3
BMI (*x* ± *S*, kg/m^2^)	24.39 ± 1.73	24.63 ± 1.51
Years of education (*x* ± *s*, years)	7.13 ± 3.33	5.16 ± 2.03
Family history of CHF (case (%))	20.9	21.4
Average annual household income (*x* ± *s*, 10,000 yuan)	3.50 ± 1.39	4.33 ± 1.66

**Table 2:** Comparison of intraoperative and postoperative clinical indexes (*x* ± *s*).

Group	*n*	Operation time (h)	Postoperative recovery time (h)	Cost of treatment (yuan)	LVEF score (%)
A group	306	19.86 ± 9.30	34.76 ± 12.01	47350.650 ± 449.35	39.21 ± 5.06
B group	337	19.65 ± 9.32	34.58 ± 12.11	47342.50 ± 429.18	40.25 ± 5.98
*t*		0.286	0.189	0.237	2.368
*P* value		0.775	0.850	0.813	0.018

**Table 3:** Comparison of MMSE score and MoCA score (*x* ± *s*, points).

Group	*n*	MMSE score		MoCA score	
		Before operation	After operation	Before operation	After operation
A group	306	22.65 ± 0.13	27.96 ± 0.46	22.80 ± 3.70	28.48 ± 5.53
B group	337	22.64 ± 0.19	26.75 ± 0.39	22.95 ± 2.86	27.52 ± 4.89
*t*		0.771	36.076	0.578	2.336
*P* value		0.441	＜0.001	0.563	0.020

**Table 4:** Comparison of HAMA score and HAMD score (*x* ± *s*, points).

Group	*n*	Before operation		After operation	
		HAMA score	HAMD score	HAMA score	HAMD score
A group	306	24.69 ± 5.03	25.36 ± 5.69	17.03 ± 5.36	21.50 ± 6.36
B group	337	24.34 ± 0.19	26.75 ± 0.39	16.95 ± 2.86	20.52 ± 4.89
*t*		1.276	4.473	2.142	2.201
*P* value		0.202	＜0.001	0.153	0.028

**Table 5:** Study on the influence of related indexes on the cognitive function of patients in A group.

Variable	Constant	*P* value	OR	90% CI
Hypertension	−0.867	0.243	0.542	0.147–1.589
FPG	0.154	0.002	1.204	0.945–1.305
HbA1c	0.201	0.025	1.299	0.883–1.561
HCY	0.049	0.374	0.215	0.518–1.097
HDL-C	−2.511	0.003	0.102	0.025–0.338

OR value: odds ratio. OR value >1 indicates that this factor is a risk factor. OR value <1 indicates that this factor is a protective factor. 90% CI： 90% confidence interval; FPG: fasting blood glucose; HbA1c: glycosylated hemoglobin; HDL-C: high density lipoprotein cholesterol; HCY： homocysteine.

## Data Availability

The data used to support the findings of this study are available from the corresponding author upon request.
